# The Effect of Inhalation Aromatherapy and Music Therapy on Anxiety in Patients Undergoing Shockwave Lithotripsy: A Randomized Controlled Clinical Trial

**DOI:** 10.1155/2022/8015798

**Published:** 2022-06-29

**Authors:** Mohammad Rohi Ganji, Faranak Jafari, Shahab Rezaeian, Hossein Abdi, Mohammad Hussein Farzaei, Alireza Khatony

**Affiliations:** ^1^Student Research Committee, Kermanshah University of Medical Sciences, Kermanshah, Iran; ^2^School of Nursing and Midwifery, Kermanshah University of Medical Sciences, Kermanshah, Iran; ^3^School of Health, Kermanshah University of Medical Sciences, Kermanshah, Iran; ^4^School of Medicine, Kermanshah University of Medical Sciences, Kermanshah, Iran; ^5^Pharmaceutical Sciences Research Center, Health Institute, Kermanshah University of Medical Sciences, Kermanshah, Iran; ^6^Social Development and Health Promotion Research Center, Health Institute, Kermanshah University of Medical Sciences, Kermanshah, Iran; ^7^Infectious Diseases Research Center, Kermanshah University of Medical Sciences, Kermanshah, Iran

## Abstract

Patients undergoing shock wave lithotripsy (SWL) have a high level of anxiety. This study was aimed to compare the effect of music therapy and aromatherapy on patients' anxiety levels during SWL. In this clinical trial, 176 patients undergoing SWL were randomly assigned to four groups: music therapy, aromatherapy, combined music therapy and aromatherapy, and control. The state-trait anxiety inventory (STAI) was used to collect data. In the aromatherapy group, three drops of rosemary essential oil were used during SWL. For the music therapy group, soft music was played during SWL. In the music therapy and aromatherapy group, soft music and three drops of rosemary essential oil were used simultaneously. In the control group, three drops of aromatic distilled water were used. The results showed that all patients had moderate anxiety before the intervention. The analysis of variance test did not show a statistically significant difference between the groups, but this difference was significant after the intervention. The levels of anxiety after the intervention were higher in the music therapy, aromatherapy, and combined music therapy and aromatherapy groups than in the control group. The results of the paired *t*-test showed the level of anxiety after the intervention was significantly increased in the intervention group (*P* < 001). In conclusion, the results indicated that music therapy, aromatherapy, and combined music therapy and aromatherapy had no effect on reducing patients' anxiety during SWL.

## 1. Introduction

Shock wave lithotripsy (SWL) is a common and effective treatment for urinary tract stones [1]. Patients experience high anxiety during SWL due to the pain of this procedure and the sounds of the device [2]. Today, anxiolytics are used to reduce anxiety, which is not highly recommended due to side effects such as hypotension and respiratory depression [2, 3]. Therefore, several nonpharmacological methods, including music, aromatherapy, hypnosis, relaxation, biofeedback, and reflexology, have been proposed to control anxiety [1]. Among these methods, music therapy and aromatherapy have been widely used due to their sedative benefits [1, 3, 4].

Aromatherapy is the therapeutic use of essential oils extracted from plants, which is a cheap and noninvasive method with relatively low complications [5]. One of the essential oils used in aromatherapy is rosemary essential oil, with the scientific name *Rose damascena* [6]. This essential oil is used to reduce anxiety, depression, and stress due to its soothing and hypnotic properties [7, 8]. The main components of rosemary essential oil include geraniol, citronellol, phenethyl alcohol, nonadecane, ethanol, nerol, heneicosane, and Kaempferol, which have provided medicinal properties to this plant [9]. The scent of rosemary essential oil transmits signals to the olfactory system and stimulates the secretion of brain neurotransmitters such as serotonin and dopamine, thereby affecting a person's emotions [10, 11].

Another method of complementary medicine is music therapy [12]. This method has become increasingly popular in the treatment of anxiety due to its low cost, availability, and high acceptance [13]. Music causes a pleasant sensation by reducing cortisol and hypothalamic-pituitary-adrenal axis neuropeptides and subsequent releasing of endorphins from the limbic system. Music also reduces amygdala activity in the brain, thereby reducing anxiety [14]. There have been several studies on the effects of aromatherapy with rosemary essential oil and music therapy on patients' anxiety levels. Some of these studies have reported that aromatherapy has no effect on anxiety levels [15–17], but some other studies have shown a positive effect [18–21]. Regarding music therapy, the results of some studies indicate the effectiveness of this method in reducing anxiety [22]. However, some other studies have reported no positive effect [23, 24].

Regarding the combined use of aromatherapy and music therapy, the results of a study indicated that this method reduced patients' anxiety, but music therapy had a higher effect than aromatherapy [25]. However, Fenko and Loock reported that combined music therapy and aromatherapy had no effect on the level of anxiety in patients waiting for surgery [26].

Considering the mentioned contradictions and also the paucity of studies that have compared the effects of two methods of inhaled aromatherapy with rosemary essential oil and music therapy on the anxiety of patients undergoing SWL, the present study was performed to shed more light on this lacuna.

This study sought to answer the following questions: (1) Is aromatherapy effective in reducing participants' anxiety in SWL? (2) Is music therapy effective in reducing participants' anxiety in SWL? and (3) Are combined music therapy and aromatherapy effective in reducing participants' anxiety in SWL?.

## 2. Materials and Methods

### 2.1. Study Design

This randomized controlled clinical trial with a parallel design and a 1 : 1 allocation ratio in the experimental (including three groups of aromatherapy, music therapy, and combined music therapy and aromatherapy therapy) and control groups was carried out based on CONSORT criteria (Reporting Randomized, Controlled Trials of Herbal Interventions: an elaborated CONSORT statement, and Reporting Guidelines for Music-based Interventions) [27, 28] and lasted from December 2020 to September 2021.

### 2.2. Study Hypothesis

The combination of aromatherapy and music therapy can reduce the state anxiety in patients undergoing SWL.

### 2.3. Sample and Sampling Method

The study population comprised all patients with kidney stones referred to the SWL unit of Imam Reza Hospital in Kermanshah-Iran. Using the estimates of a previous study [27] with a mean difference of 2.04 in the control group and a difference of 1.7 and a standard deviation of 0.45 at 95% confidence level, the sample size was estimated to be 176 patients, 23 patients in each group. To detect the effect of interaction, the sample size was increased by 50%, and by applying a 20% drop and noncooperation, the sample size was increased to 44 patients in each group. The samples were recruited by the convenience sampling method and were randomly assigned to the study groups using 8-item randomized blocking. Random blocking was created using the website https://www.sealedenvelope.com. The person collecting the data as well as the person analyzing the data were unaware of the type of sample allocation to the study groups.

The following were considered for the random allocation process: (A) blocks of 8 were considered; (B) one letter was assigned to each of the groups (A to the music group, B to the aromatherapy group, C to the combined music and aromatherapy, and D to the control group); (C) a sequence was created for a sample size of 200; and (D) for the random allocation concealment process, 25 opaque envelopes and 200 cards were created. Inside each envelope, eight cards were placed in sequence. The number of blocks was written on each envelope. On each card, the name of the desired group was written in sequence. The inclusion criteria were: willingness to participate in the study, age range of 18–65 years, no history of any allergies (because allergy is one of the side effects of essential oils [29]), no respiratory diseases, having a healthy sense of smell and hearing, no drug addiction, no thyroid disease, stable vital signs, no history of psychiatric illness, and no use of psychotropic drugs. In order to assess the health of the sense of smell, the openness of the nostrils was examined. Further, a cardamom seed was placed separately in front of each nostril, and if correctly diagnosed, it showed olfactory health. The exclusion criteria included receiving drugs and antianxiety drugs during the study and the patient's unwillingness to continue participation in the study for any reason.

### 2.4. Instruments

The STAI was developed by Spielberger (1983) to measure the state and trait anxiety [30]. This tool has been psychometrically investigated in previous studies (Cronbach's alpha coefficient = 0.86) [31]. The Persian version of STAI has been psychometrically analyzed in Iran, with its internal consistency being determined by Cronbach's alpha (0.88) [32]. The STAI has two scales, including state and trait anxiety. In this study, state anxiety was examined, which includes twenty items. The answers are based on a four-point Likert scale, including very low (1), low (2), high (3), and very high (4). The STAI score ranges from 20 to 80, and patients fall into one of the three categories according to their score, including mild anxiety (20 to 39), moderate anxiety (40 to 59), and severe anxiety (60 to 80).

In this study, the Lander LD-30 MP3 Player (made in China) was used to play the music. Lenovo LivePods wireless headphones (made in China) were also used to listen to music. It should be noted that the name of the SWL machine was STORZ SLX 2001.

### 2.5. Interventions

In the current trial, all patients enrolled in the study were elective. When patients with urolithiasis were referred to a urologist (fourth author), they were provided with the necessary written and oral training. The date of the patients' referral for SWL was determined by the office secretary. In the morning of the procedure, the necessary tips were given to patients by the nurse of the SWL unit, and their questions were answered. It should be noted that SWL procedures were performed by a urologist (fourth author). In the current study, after obtaining approval from the university ethics committee, the researcher was referred to the SWL unit of Imam Reza Hospital. This hospital is the largest subspecialty center in Western Iran. First, the objectives of the study were described to the patients, and if they were willing, they were recruited in the study. In the next step, the patients were randomly assigned to one of the four study groups, including music, aromatherapy, combined music and aromatherapy, and control. Thirty minutes before the intervention, the demographic information form and STAI were completed by all patients. In the music therapy group, traditional soft music was played using an MP3 player 15 minutes before and during the SWL. The name of the song was Golnoosh, composed by Parviz Meshkatian, a famous Iranian composer. Patients were asked to calmly focus on the music being played. In the aromatherapy group, rosemary essential oil with 25% purity was used 15 minutes before and during SWL. The essential oil was made by Zarband-Iran Pharmaceutical Company and was stored in dark containers, away from light and heat, at a temperature of 2–8°C. To perform the intervention, 3 drops of rosemary essential oil were dropped on a cotton ball and attached to the collar of the dress, and the patient was asked to breathe normally. In the third group, a combination of music and aromatherapy was used. For this purpose, three drops of 25% rosemary essential oil and soft traditional music (Golnoosh song) were used simultaneously. In the control group, three drops of aromatic distilled water were used. Immediately after SWL, the STAI was completed again by the samples in all four groups. In the current study, due to the nature of the interventions, it was not possible to blind patients, and blindness was only done for the statistical consultant of the study as he was not aware of the names of the groups. It should be noted that there was no dropout in any of the four groups, and all patients were included in the analysis phase. The study process is shown in Figure 1.

### 2.6. Data Analysis

Data were analyzed by SPSS software (SPSS v.18.0; SPSS Inc., Chicago, IL, USA) using descriptive (mean, frequency, and standard deviation) and inferential (paired *t*-test, one-way analysis of variance (ANOVA), and repeated measures ANOVA) statistics. The ANOVA test was used to examine the homogeneity of variables in the four study groups and to compare the mean anxiety of the study groups before and after the intervention. The paired *t*-test was performed to compare the mean anxiety levels in each study group before and after the intervention. Repeated measures ANOVA was applied to evaluate the effects of aromatherapy, music therapy, combined music therapy and aromatherapy, and the interaction of two factors: STAI time (before and after the intervention) and the intervention group. The level of significance for all tests was less than 0.05.

### 2.7. Ethical Considerations

The study was based on the Declaration of Helsinki. The ethics committee of Kermanshah University of Medical Sciences approved the study (No: IR.KUMS.REC.1399.651). The study was also registered in the Iranian Registry of Clinical Trials database under the number IRCT20100913004736N23. The objectives of the study were explained to all samples, and written informed consent was obtained from them. All samples were assured that their information and responses would be kept confidential.

## 3. Results

A total of 176 patients with kidney stones were assigned to one of four groups: aromatherapy, music therapy, combined aromatherapy and music therapy, and control (44 patients in each group). The mean age of the samples was 41 years. Most of the samples were male (64.2%, *n* = 113), married (78.4%, *n* = 138), undergraduate (76.1%, *n* = 134), and nonsmoking (82.3%, *n* = 145). About half of the samples had no history of SWL (52.3%, *n* = 92) and 66.3% (*n* = 112) had urine stones of 20–20 mm. All four groups were homogeneous in terms of demographic variables (Table 1).

The mean anxiety scores before and after the intervention were 45.8 ± 2.5 and 47.5 ± 2.2 out of 63 in the aromatherapy group (*P*=0.003), 46.0 ± 3.2 and 48.2 ± 2.0 in the music therapy group (*P* < 0.001), 45.7 ± 3.1 and 47.9 ± 2.3 in the combined aromatherapy and music therapy group (*P*=0.001), and 46.5 ± 3.8 and 45.9 ± 3.5 in the control group, respectively (*P*=0.244). The results of the ANOVA test showed no statistically significant difference between the study groups in terms of mean anxiety before the intervention, but this difference was statistically significant after the intervention (*P* < 0.001). The results of a paired *t*-test showed a statistically significant difference between the mean anxiety scores before and after the intervention in the music therapy, aromatherapy, and combined aromatherapy and music therapy groups, but this difference was not significant for the control group (Table 2).

The results of the repeated measures ANOVA test showed that considering the effect of group and intervention, the effect of time on mean anxiety had a significantly increasing trend (*P* < 0.001, *F* = 23.983). Further, the effect of the intervention was significant considering the effect of time and group (*P*=0.001, *F* = 5.678). In addition, considering the effects of time and intervention, the effect of the group was not significant (Table 3).

## 4. Discussion

This study aimed to compare the effects of inhalation aromatherapy with rosemary essential oil and music therapy on the level of anxiety in patients undergoing SWL. The results showed aromatherapy with rosemary essential oil had no effect on patients' anxiety levels. In this regard, the results of a clinical trial showed that aromatherapy had no effect on the anxiety level of patients admitted to the Intensive Care Unit (ICU) [17]. However, a clinical trial on the effect of aromatherapy with rosemary essential oil and progressive muscle relaxation technique on the anxiety level of 90 patients undergoing general surgery showed that these two methods to some extent reduced patients' anxiety [33]. Increased patient anxiety during SWL is not unexpected because it is a painful and stressful intervention [2]. Part of this stress is related to the device sounds and fear of treatment failure [2, 23]. Among the reasons for the ineffectiveness of aromatherapy in the present study are the high level of patients' anxiety, the short duration of the intervention, and the lack of attention to patients' opinions while choosing the type of aroma.

In the present study, music therapy had no effect on patients' anxiety levels during SWL. In this regard, the results of a clinical trial performed on 300 patients undergoing SWL showed that music had no effect on anxiety levels [34]. Another study on the effects of stress bullets and music therapy on the anxiety level of 120 patients during SWL showed that these interventions were ineffective [23]. Moreover, a clinical trial on the effect of music on anxiety levels in 102 patients undergoing radiotherapy indicated that music had no effect on anxiety [24]. In addition, a clinical trial on the effect of different kinds of music, including folk, soft, and classical, on anxiety levels among 200 patients undergoing SWL revealed that music could reduce the patients' anxiety [2]. SWL is a stressful intervention that is associated with patient pain and anxiety and sometimes requires medical intervention [1, 2]. Regarding the reasons for the ineffectiveness of music in the current study, we can mention the short duration of the intervention, the stressful nature of the SWL, and the lack of attention to patients' opinions when choosing the type of music.

In the present study, the combined music therapy and aromatherapy had no effect on anxiety levels. So far, no study has been performed on the combined use of music and aromatherapy on patients undergoing SWL. A clinical trial was conducted to compare the effects of ambient odor and music on the level of anxiety in waiting room patients. A total of 117 patients were randomly allocated to one of four groups: no scent-no music condition, scent condition, scent-music condition, and music condition. Eight different types of fragrances such as vanilla, lavender, rose, magnolia, and mango were used. Three types of music were played to the patients' choice. The results showed that the combination of music and aroma in the environment had no effect on patients' anxiety levels [26]. A clinical trial comparing the effects of music and massage aromatherapy on the anxiety levels of 132 patients under mechanical ventilation showed the effectiveness of these two methods in reducing anxiety [25]. Several factors affect the effectiveness of music therapy and aromatherapy, including the patients' opinions in choosing the type of music and aroma, the length of the intervention, and the elimination of stressors in the patient's room [2, 25, 26]. Although in the present study the researchers tried to minimize the impact of environmental factors on patients' anxiety, factors such as lack of previous SWL experience and disregard for patients' opinions on choosing the type of music and aroma might have reduced the effectiveness of music therapy and aromatherapy.

### 4.1. Study Limitations

This study faced several limitations. The main limitation was the impossibility of performing gas chromatography-mass spectrometry (GC-MS) for financial reasons. However, Zarband Pharmaceutical Company is a reputable company approved by the Ministry of Health of Iran. Another limitation was the nonselectivity of the type of music or fragrance used, which could have affected the results of the study. The mental state of the participants while completing the STAI might have affected their answers to the questions. The last limitation is that soft traditional music used to reduce anxiety levels may cause different reactions in patients from other countries, with other musical habits and traditions.

## 5. Conclusion

This clinical trial compared the effects of aromatherapy, music therapy, and combined aromatherapy and music therapy on the patients' anxiety during SWL. The results showed that all of these interventions were ineffective. The ineffectiveness of these interventions can be indicated by the patients' high level of anxiety, the short duration of the interventions, and a lack of attention to the patients' opinions on choosing the type of music and aroma. Future studies are recommended to increase the duration of these interventions to at least one hour before the start of SWL. Future studies are also suggested to choose the type of music and aroma based on the patients' opinions.

## Figures and Tables

**Figure 1:** The CONSORT diagram of the study.

**Table 1:** Demographic characteristics of patients.

Variables		Groups				*P* value
		Aromatherapy	Music therapy	Combined aromatherapy and music therapy	Control	
Gender	Male	32 (77.7)	24 (54.5)	28 (63.6)	27 (61.4)	0.398
	Female	12 (27.3)	20 (45.5)	16 (36.4)	17 (38.6)	
Age (years) (mean ± SD^†^)	—	46.0 ± 11.5	42.8 ± 12.2	44.3 ± 10.7	44.0 ± 13.5	0.908
BMI^ǁ^ (mean ± SD)	—	26.3 ± 4.2	25.6 ± 3.3	27.0 ± 3.8	25.7 ± 3.8	0.352
Marital status	Single	9 (20.4)	12 (27.2)	7 (15.9)	12 (27.3)	0.591
	Married	35 (79.6)	32 (72.8)	37 (84.1)	32 (72.7)	
Education	Nonacademic^††^	32 (72.7)	30 (68.2)	36 (81.8)	36 (81.8)	0.769
	Academic	12 (27.3)	14 (21.9)	8 (18.2)	8 (18.2)	
Smoking	Yes	12 (27.3)	8 (18.2)	8 (18.1)	7 (16.0)	0.811
	No	32(72.7)	36 (81.8)	36 (81.9)	37 (84.0)	
Stone size (mm)	<10	9 (20.4)	11 (25.0)	15 (34.1)	15 (34.0)	0.086
	11–20	29 (65.9)	29 (65.9)	26 (59.0)	26 (59.2)	
	>21	6 (16.6)	4 (9.1)	3 (6.9)	3 (6.8)	
Stone location	Renal pelvis	13 (29.5)	14 (31.8)	16 (36.4)	15 (34.1)	0.845
	Calyx	22 (50.0)	19 (43.2)	20 (45.5)	19 (43.2)	
	Upper ureteral	9 (20.5)	11 (25.0)	8 (18.2)	9 (20.5)	
	Middle ureteral	—	—	—	1 (2.3)	
Stone laterality	Right	18 (40.1)	23 (52.3)	22 (50.0)	17 (38.6)	0.334
	Left	26 (59.9)	21 (47.7)	22 (50.0)	27 (61.4)	
Previous history of SWL^*θ*^	Yes	21 (47.7)	22 (50.0)	23 (52.3)	22 (50.0)	0.549
	No	23 (52.3)	22 (50.0)	21 (47.7)	22 (50.0)	
ESWL duration (min) (mean ± SD)	—	26.2 ± 1.9	25.6 ± 2.4	25.3 ± 3.1	25.5 ± 2.5	0.384
ESWL energy (j) (mean ± SD)	—	7.9 ± 0.3	7.9 ± 0.3	7.7 ± 0.5	7.7 ± 0.5	0.041^§^
Number of ESWL blows (mean ± SD)	—	2333.7 ± 146.8	2285.7 ± 204.3	2251.3 ± 254.7	2284.1 ± 207.9	0.304

*Note*: ^†^ standard deviation, ^ǁ^ body mass index; ^*θ*^ extracorporeal shock wave lithotripsy; ^‡^ nonsignificant; ^††^ high school diploma and less than high school. ^§^ The difference is significant at *P* < 0.05.

**Table 2:** Comparison of mean state anxiety before and after intervention in study groups.

Groups	Before		After		*P* value		
	Mean	95% CI	Mean ± SD	95% CI	Time	Time × group	Group
Aromatherapy	45.8 ± 2.5	44.8, 46.7	47.5 ± 2.2	46.8, 48.3	0.032	<0.001^§^	<0.001^§^
Music therapy	46.0 ± 3.2	45.1, 47.0	48.2 ± 2.0	47.4, 49.0			
Combined aromatherapy and music therapy	45.7 ± 3.1	44.8, 46.7	47.9 ± 2.3	47.1, 48.6			
Control	46.5 ± 3.8	45.6, 47.5	45.9 ± 3.5	45.1, 46.7			
Test result	*F* = 0.577, *P*=0.631		*F* = 6.765, *P* < 0.001^§^				

*Note.* The results of ANOVA test showed no statistically significant difference between the study groups in terms of mean anxiety before the intervention, but this difference was statistically significant after the intervention. The results of paired *t*-test showed a statistically significant difference between the mean anxiety scores before and after the intervention in the music therapy, aromatherapy, and combined aromatherapy and music therapy groups, but this difference was not significant in the control group. ^§^The difference is significant at *P* < 0.05.

**Table 3:** Comparison of mean state anxiety before and after intervention in study groups.

Groups	Pretest	Post-test	Difference (post-pre)	Test results
	Mean ± SD	Mean ± SD	Mean ± SD	
Aromatherapy	45.8 ± 2.5	47.5 ± 2.2	1.7 ± 3.8	*t* = 3.104, *P*=0.003^§^
Music therapy	46.0 ± 3.2	48.2 ± 2.0	2.2 ± 3.6	*t* = 3.896, *P* < 0.001^§^
Combined aromatherapy and music therapy	45.7 ± 3.1	47.9 ± 2.3	2.2 ± 3.9	*t* = 3.656, *P*=0.001^§^
Control	46.5 ± 3.8	45.9 ± 3.5	−0.6 ± 3.4	*t* = −1.181, *P*=0.244
Test results	*F* = 0.577, *P*=0.631	*F* = 6.765, *P* < 0.001^§^		

*Note.* Considering the effect of group and intervention, the effect of time on mean anxiety had a significantly increasing trend. Further, the effect of the intervention was significant considering the effect of time and group. In addition, considering the effect of time and intervention, the effect of the group was not significant. ^§^The difference is significant at *P* < 0.05.

## Data Availability

The identified datasets analyzed during the current study are available from the corresponding author upon a reasonable request.
